# Emotion Recognition Based on EEG Using Generative Adversarial Nets and Convolutional Neural Network

**DOI:** 10.1155/2021/2520394

**Published:** 2021-10-11

**Authors:** Bo Pan, Wei Zheng

**Affiliations:** School of Electronics and Information, Jiangsu University of Science and Technology, Zhenjiang 212100, China

## Abstract

Emotion recognition plays an important role in the field of human-computer interaction (HCI). Automatic emotion recognition based on EEG is an important topic in brain-computer interface (BCI) applications. Currently, deep learning has been widely used in the field of EEG emotion recognition and has achieved remarkable results. However, due to the cost of data collection, most EEG datasets have only a small amount of EEG data, and the sample categories are unbalanced in these datasets. These problems will make it difficult for the deep learning model to predict the emotional state. In this paper, we propose a new sample generation method using generative adversarial networks to solve the problem of EEG sample shortage and sample category imbalance. In experiments, we explore the performance of emotion recognition with the frequency band correlation and frequency band separation computational models before and after data augmentation on standard EEG-based emotion datasets. Our experimental results show that the method of generative adversarial networks for data augmentation can effectively improve the performance of emotion recognition based on the deep learning model. And we find that the frequency band correlation deep learning model is more conducive to emotion recognition.

## 1. Introduction

Emotions are fundamental in the daily life of human beings as they play an essential role in human cognition, namely, in perception, rational decision-making, human interaction, and human intelligence [1]. With the development of artificial intelligence technology and deep learning, emotion recognition has broad prospects in human-computer interaction and clinical treatment, which has been widely concerned by researchers [2].

Human emotions can be recognized by speech, eye blinking, facial expressions [3–5], and physiological signals [6]. However, the first three methods are unstable and easily affected by subjectivity. Subjects can deliberately conceal their emotions and lead to recognition errors. Physiological signals such as electrooculogram (EOG), electroencephalogram (EEG), and blood pressure (BVP) are produced spontaneously by the human body. Therefore, physiological signals can more accurately reflect the emotional state of people. Among all these physiological signals, electroencephalogram (EEG) is the overall reflection of the electrophysiological activities of brain nerve cells on the cerebral cortex or scalp surface, which indicates that changes in EEG signals can be used to characterize human emotional changes.

Due to the advantages of EEG in reflecting emotions, an EEG signal has been widely used for the research on emotion recognition [7–10]. The changes in scalp potential are captured by multiple electrodes. Once the subject is stimulated, the brain electrodes can immediately capture the potential changes to identify the emotional state. There are two general rules to classify human emotions, namely, the discrete basic emotion description and the dimensional method. According to the discrete basic emotion description method, emotions can be divided into six basic emotions, including joy, surprise, sadness, fear, anger, and disgust [11]. For dimensional methods, emotions are usually divided into two dimensions (arousal and valence). Among these dimensions, arousal describes an emotion's level of excitement or apathy, and valence describes a person's level of positivity or negativity. Compared with discrete basic emotion description, the dimensional method is simpler, so the dimensional method is often used in emotion recognition [12]. An early work on emotion recognition by analyzing EEG signals dates back more than 50 years [13]. Recently, many new feature extraction and classification methods have been proposed for emotion recognition [14]. In the feature extraction stage, the time-domain method, frequency-domain method, and nonlinear dynamic method are often used to analyze EEG signals. For example, time-domain analysis can extract the time-dependent features of EEG signals, including sample entropy, statistical features, and principal component analysis [15]. In frequency-domain analysis, EEG signals can be broken down into *δ* (1-3 Hz), *θ* (4-7 Hz), *α* (8-13 Hz), *β* (14-30 Hz), and *γ* bands (31-50 Hz); features can be extracted from each frequency band [16, 17].

In recent years, many researchers have built emotion recognition models based on machine learning. Chanel and others used EEG signals. Time-frequency information was extracted as the feature, and a Support Vector Machine (SVM) was used as the classifier to distinguish three kinds of emotional states [18]. Heraz and Frasson used the amplitude of the EEG signal as the feature and divided human emotional states into eight categories by *k*-Nearest Neighbors (KNN) [19]. Currently, deep learning has been widely used in the field of EEG emotion recognition. Zheng and Lu studied the influence of various frequency bands on emotion recognition through neural networks and concluded that the *β* and *γ* frequency bands are more suitable for EEG emotion recognition tasks [6]. A recent study also confirmed that the high-frequency band can better distinguish emotional states [20]. Tang et al. used recurrent neural networks and autoencoders to classify emotional states, which greatly improved the accuracy of EEG emotion recognition and achieved an average accuracy of 83.25% [21]. Xiang et al. adopted a new preprocessing method, instead of using one-dimensional data like traditional methods, but converting EEG signals into 2D frames and combining convolutional neural networks (CNN) and recurrent neural networks for emotional state recognition [22]. Li et al. extracted the Power Spectral Density (PSD) feature and mapped its one-dimensional feature vector to a two-dimensional plane to construct a feature map using convolutional neural networks and long-short-term memory networks to identify human emotional states [23]. Generally speaking, researchers of EEG emotion recognition based on deep learning mostly map EEG signals into pictures to facilitate input into neural networks. They encapsulate the data into a similar image and then use a convolutional neural network to obtain higher accuracy [24–28].

Based on the excellent performance of deep learning in the EEG emotion recognition task, it is necessary to use the deep learning model to promote the exploration of EEG-based emotion recognition. However, the deep learning model is data-driven, and only when there are many data can it have good performance, which makes the training of a deep learning model need a large number of labeled training samples. However, due to the high cost, most public EEG datasets have only a small number of samples, and these sample categories are extremely unbalanced. Insufficient sample size and unbalanced categories will lead to overfitting and seriously affect the performance of the deep learning model. Therefore, if we try to further explore the deep learning model of emotion recognition based on EEG signals, obtaining enough effective marker training data is the main problem.

In this paper, we focus on generating more EEG training samples through the data augmentation method of generative adversarial networks to solve the imbalance between sample categories. After that, we explore the performance of emotion recognition with the frequency band correlation and frequency band separation computational models before and after data augmentation on standard EEG-based emotion datasets.

## 2. DEAP Dataset

DEAP [29] (Database for Emotion Analysis using Physiological Signals) is the database collected by Koelstra from Queen Mary University of London; the University of Twente; the University of Geneva, Switzerland; and the Swiss Federal Institute of Technology. Multichannel data are for studying human emotional states. At present, the DEAP dataset has been widely used in emotion recognition research. Therefore, in this paper, we use this dataset to test our method. The database is based on the physiological signals generated by the stimuli induced by music video materials. It recorded 32 subjects who watched 40 minutes of music videos (1 minute for each music video) of physiological signals and the subjects' self-assessment on valence and arousal. Arousal and valence scales are from 1 to 9 (1 represents sad/calm and 9 represents happy/excited). The sampling rate of physiological signals is 512 Hz. For researchers to quickly verify their proposed emotion recognition method, the creator of the DEAP dataset provided a preprocessed version of the dataset. In the preprocessed dataset, the original EEG signal is downsampled from 512 Hz to 128 Hz, only the signal in the 4–45 Hz frequency bandwidth is preserved, and the EOG is also removed. The data collected in each trial was segmented into 3-second pretrial baseline signals (relax state) and 60-second experimental signals (recorded while watching a video). The EEG data for each participant includes two arrays: data and labels. Tables 1 and 2 show a summary of the DEAP dataset (preprocessed version).

## 3. Methods

### 3.1. Data Preprocessing

Based on the in-band correlation with different behavioral states, the original EEG signal can be divided into several different frequency modes [30–32]. According to Zhang et al. [33], the EEG frequency, mode, and corresponding characteristics are shown in Table 3. It can be found from the table that the recognition increases with the increase in the frequency band. Therefore, to identify emotions more accurately, we only use *θ*, *α*, *β*, and *γ*, which represent the frequency band when human thinking is active.

The brain-computer interface system for capturing brain electrical signals uses a wearable headset device with multiple electrodes. The 10-20 system electrode placement method is the standard electrode placement method prescribed by the International Electroencephalography Society. In addition, the “10” and “20” in the international 10-20 system refer to the distance from the midpoint of the frontal pole to the root of the nose and the distance from the occipital point to the extra occipital tuberosity accounting for 10% of the total length of the line. Points are separated by 20% of the total length of this line. The left picture of Figure 1 is a plan view of the international 10-20 system, in which the yellow-filled EEG electrodes are the test points used in the DEAP dataset. In the EEG electrode map, there is a spatial position connection between the electrodes. To reflect the spatial position information between the electrodes, we map the one-dimensional EEG data to a two-dimensional plane according to the spatial position relationship of the electrodes. At the same time, the unused electrodes are filled with 0. The right image of Figure 1 shows the two-dimensional plane after mapping.

For the original 63-second EEG data, we removed the baseline part of the first 3 seconds and only retained the 60-second experimental data. EEG data of a participant were converted from 40 × 32 × 8064 to 40 × 32 × 7680. To increase the amount of training data, we divide the EEG data segment into multiple samples, each of which has a length of 2 seconds, of which 1 second overlaps, and assign every sample with the label of the original trial (step 1). Next, feature extraction is performed on all samples. First, we use the Butterworth filter to decompose each sample into three frequency bands *θ*, *α*, *β*, and *γ* (step 2). Secondly, we extract PSD features and normalize each PSD vector with *Z*-score normalization (step 3). Thirdly, we organize the PSD feature of each frequency band as a 2D map (step 4) and stack them (step 5). The whole process is described in Figure 2. PSD is widely applied in most EEG-based tasks and is considered one of the most commonly used features, which is defined as

(1) $$\begin{array}{c} P\left(\omega_{i}\right)=\frac{1}{N}{\left|X\left(\omega_{i}\right)\right|}^{2}. \end{array}$$

The discrete Fourier transform *X*(*ω*_*i*_) of the signal can be obtained by FFT, where *ω*_*i*_ is the frequency point of the number *i*.

### 3.2. Data Augmentation Method

In EEG emotion recognition tasks, most methods rely on sufficient sample data and the balance between sample classes. However, in actual experiments, many datasets do not meet such requirements. For example, after the DEAP dataset used in this experiment is processed in Figure 2, the ratio of high arousal to low arousal is 4 : 1 or 4 : 3 for most individuals, but only a small proportion is 1 : 1, and the overall data sample is unbalanced. The traditional methods that are used to solve the problem of sample imbalance can be classified into sample sampling and improved recognition models. Among them, sample sampling is divided into two types: oversampling [34] and undersampling [35]. Oversampling generates duplicate samples through copy operation, which will cause the classifier to overfit; undersampling technology eliminates some large samples, and the information may be serious. The loss leads to the distortion and incompleteness of the information space. The way to improve the recognition model starts from the recognition model itself and often improves the recognition accuracy by adjusting the sensitivity of the classifier. The degree of improvement is often limited, and it is difficult to obtain the optimal weight.

Goodfellow et al. [36] proposed a semisupervised feature learning algorithm based on game scenes in 2014-Generative Adversarial Networks (GAN) to improve this limitation. With the continuous improvement of adversarial learning ideas, GAN has been applied in the fields of image generation, image recognition, and style transfer [37] and has derived variants that implement different functions. GAN learns the data distribution of training samples through the game process of generating a network and discriminating the network, so that the generator can generate very real fake samples, thereby solving the problem of an unbalanced distribution of real EEG data samples. Based on GAN, we propose Power Spectral Density Generative Adversarial Network (PSD-GAN), whose structure is shown in Figure 3.

PSD-GAN means generating samples with PSD features through GAN. First, its input is a 1 × 16-dimensional random noise. Then, a fake sample is generated by the generator. The generator consists of three linear layers and three activation functions, which are two ReLU functions and one Tanh function. Finally, the real sample and the fake sample are sent to the discriminator for identification. The discriminator structure is composed of two linear layers and two activation functions, that is, a LeakeReLU function and a sigmoid function. Note that the real sample here is not a 3D frame but a 1 × 128-dimensional vector that is converted from the 1 × 32 × 4-dimensional vector in step 3 of Figure 2. The whole process optimizes the cost function through continuous repeated training. Details of the cost function as follows:

(2) $$\begin{array}{c} \underset{G}{\min}\underset{D}{\max}V\left(D,G\right)=E_{x\sim p_{\text{data}}\left(\text{x}\right)}\left[\log\left(D\left(x\right)\right.\right]+E_{\text{z}\sim p_{z}\left(z\right)}\left[\log\left(1-D\left(G\left(z\right)\right)\right)\right]. \end{array}$$

In this cost function, *D*(*x*) represents the discrimination of real samples and *G*(*z*) represents the generated samples. *G* hopes that *D*(*G*(*z*)) is as large as possible; at this time, *V*(*D*, *G*) will become smaller. *D* hopes that *D*(*x*) should be larger and *D*(*G*(*z*)) should be smaller. At this time, *V*(*D*, *G*) will become larger. Through such continuous alternating training, a Nash equilibrium will eventually be reached. After the training is completed, we convert the generated sample 1 × 128-dimensional vector into a 3D frame through steps 4 and 5 in Figure 2.

### 3.3. Frequency Band Correlation and Frequency Band Separation Models

CNN has a powerful function of extracting features from images. It has become a common practice for most researchers to encapsulate EEG data in the form of 3D frames and use the functions of CNN for feature extraction.

To explore the influence of the correlation features between frequency bands on the accuracy of EEG signal emotion recognition, two comparisons Frequency Band Correlation Convolutional Neural Network (FBCCNN) and Frequency Band Separation Convolutional Neural Network (FBSCNN) are designed. The essential difference between the two models is whether CNN is used to extract features between frequency bands. The input of FBCCNN is a 3D frame, and the features extracted by the convolutional neural network contain frequency band correlation features. The input of FBSCNN is four 1D planes, which are decomposed by the 3D frames, and FBSCNN merges the features extracted by multiple 1D plane inputs before the first fully connected layer. The features extracted in this way only contain the independent features of each frequency band without frequency band correlation features. In the experiment, we keep the total number of features of FBCCNN and FBSCNN after input passing through the convolutional neural network. More details of the model are shown in Figure 4.

Both models consist of seven 2D convolutional layers, three fully connected layers, and one softmax layer. The continuous convolution method is selected between the convolutional layers; that is, there is no pooling layer between the convolutional layers. The pooling layer is to reduce the data dimension, but in the EEG emotion recognition task, because the data frame is small, the pooling layer is discarded in our model. In addition, to prevent the loss of information, a zero-filling method is used in each convolutional layer. For the size of the convolution kernel of each convolution layer, we use a 3 × 3 convolution kernel, which reduces the number of parameters while maintaining a larger receptive field, which will be more conducive to extracting feature information. After each convolutional layer, a batch normalization layer and a ReLU layer are connected. The former will make the entire neural network easier to converge, and the latter will increase the nonlinear conversion capability of the model. To increase the model expression ability between the fully connected layers, the ReLU layer is also added. The output of the fully connected layer is sent to the softmax layer to obtain the classification result. The number of feature maps in each layer of the FBCCNN model and the FBSCNN model is shown in Figure 4. It is worth noting that the number of features in each layer of the two models is roughly the same, and the difference is only reflected in the first and last convolutional layers.

## 4. Experiment

### 4.1. Experimental Setup

In our experiments, all neural networks are implemented using the PyTorch framework and trained from scratch on the Nvidia Titan RTX GPU in a fully supervised manner. For training using adaptive moment estimation (Adam), the minimum batch size is 64 EEG streams. The learning rate is 0.0001, and the number of training is 150 epochs.

As mentioned above, we use the DEAP dataset to verify the performance of the proposed method. In the DEAP dataset, we select S01, S02, S04, S06, S07, S08, S09, S10, S11, S17, S18, and S22 as the experimental samples, because the positive and negative ratios of each of them are not much different. In the two-category task, for each subject, arousal and valence are divided into two categories: if the score is greater than five, the label is set to high; otherwise, it is set to low. In the four-category task, each subject is divided into four categories according to the correlation between valence and arousal: High Valence and High Arousal (HVHA), Low Valence and High Arousal (LVHA), High Valence and Low Arousal (HVLA), and Low Valence and Low Arousal (LVLA).

In subject experiments, each subject has a total of forty EEG experiments. We select the first 32 experiments as the training dataset and the last 8 experiments as the test dataset. In the across-subject experiment, all the data were shuffled. We used 80% of the data as the training dataset and 20% as the test dataset. In all comparative experiments, we use PSD-GAN to increase the training dataset samples so that the number of samples in each category is the same. This number refers to the category with the largest number in different categories. The comparison of the number of samples before and after the data augmentation of the two-category training dataset is shown in Table 4, and the comparison of the number of samples before and after the data augmentation of the four-category training dataset is shown in Table 5.

### 4.2. Experimental Results and Comparison with Different Models

To check the influence of PSD-GAN and frequency band correlation features on the classification results, we designed two scenarios, conducted experiments on the two models, and compared their results. Case 1 represents the case where PSD-GAN is not used to generate samples, and case 2 represents the case where PSD-GAN is used to generate samples. We use FBCCNN and FBSCNN to conduct a controlled experiment in each case to explore the influence of frequency band correlation features on EEG emotion recognition. A tenfold cross-validation method was used for each experiment, and the average value was calculated as the final result. The experimental result is shown in Tables 6 and 7.

As shown in Table 6, in the two classification tasks, for a single subject, the accuracy of the proposed data augmentation method in valence recognition and arousal recognition is improved by 5.25% and 6.38% on average and 6.5% and 6.71% on average across subjects. In the four classification tasks, as shown in Table 7, the data augmentation method increased by 10.92% for a single subject and 14.47% across subjects. It can be seen that the recognition accuracy has been significantly improved in two classification tasks and four classification tasks, which shows the effectiveness of this method. The data augmentation method uses the existing EEG samples in the training dataset to generate new EEG samples through the PSD-GAN network. The experimental results show that this method is useful. In addition, we can also find that before and after data augmentation, the recognition effect of the FBCCNN model is always better than FBSCNN in two classification tasks and four classification tasks, which shows that the frequency band correlation model can extract more useful features for emotion recognition than the frequency band separation model. In the experimental results, we found that there are great differences in the recognition rate of some subjects. For example, the difference between the accuracy of S07 and S22 in the arousal dichotomous task is 16.49%. These differences are mainly due to individual differences, resulting in different EEG signal intensity and responses to environmental stimuli. In addition, the improvement effect of the recognition rate before and after data augmentation in the four categories is significantly better than that before and after data augmentation in the two categories. This is because there are fewer samples added in the two categories, and the balance between samples is higher than that in the four categories, so the space for the improvement of the recognition accuracy of the two categories is less than that of the four categories. This result also shows that data augmentation is an effective way to improve the recognition accuracy in EEG emotion recognition tasks.

We also compare our model with some existing models that can identify emotions from EEG signals. Our model combines PSD-GAN and FBCCNN. We compared eight studies on emotion recognition from EEG signals, and the comparison results are shown in Figure 5. They all use the DEAP dataset for evaluation, so this comparison is meaningful. Among them, the first 4 studies employed handcrafted features and classical recognition frameworks such as Bayesian network, SVM, and HMM [37–40]. The recent 4 studies employ deep neural network architectures such as CNN and LSTM for the recognition framework [41–44]. Through comparison, it is found that our model is better than the manual feature model. Compared with other deep learning models, it also achieves better or equivalent results. However, some other deep learning models are more complex than ours. For example, the multicolumn CNN model proposed by Yang uses multiple CNN models for parallel computing and then obtains the final result by voting. Therefore, our model is highly competitive.

### 4.3. Experimental Results on the MAHNOB-HCI Dataset

The MAHNOB-HCI dataset is a multimodel dataset for emotion recognition and implicit marking, including EEG data recorded by using an EEG cap according to the international standard A 10-20 system with 32 channels. The length of the emotional video as a stimulus is between 34.9 and 117 seconds. In the experiment, we took the EEG fragments according to the valence divided into three categories, negative (1-3), neutral (4-6), and positive (7-9). There are a total of 188 negative samples, 208 neutral samples, and 131 positive samples. In Section 4.2, we have explored the impact of improving the imbalance between classes by PSD-GAN on the DEAP dataset. In this section, in order to verify our proposed PSD-GAN-extended sample and the universality of the method, we continue to experiment on the MAHNOB-HCI dataset and compare the performance difference between FBCCNN and FBSCNN.

In Table 8, we show the emotion recognition rates of two different models before and after PSD-GAN-expanded samples. For each model, our training dataset and test dataset are divided by 4 : 1. Therefore, the number of negative samples in our training dataset is 150, the number of neutral samples is 166, and the number of positive samples is 104. We used the same method of preprocessing EEG segments in the DEAP dataset for each sample and expanded the number of samples in each category to 166 through PSD-GAN.

From Table 8, we can know the details of FBCCNN and FBSCNN before and after PSD-GAN sample expansion on the MAHNOB-HCI dataset. For FBCCNN, the accuracy before and after sample expansion is improved from 62.06% to 70.34%. For FBSCNN, the accuracy before and after sample expansion is improved from 56.78% to 66.50%. In addition, we can also find that the accuracy of FBCCNN is always higher than that of FBSCNN before and after sample expansion. In the MAHNOB-HCI dataset, the results also show that the data augmentation method proposed by us can effectively improve the accuracy of emotion recognition and also confirm that the frequency band correlation model is better than the frequency band separation model.

## 5. Discussion

In this paper, we propose a new sample generation method based on the PSD-GAN network to solve the imbalance between sample categories and explore the effects of the frequency band correlation model and frequency band separation model on EEG emotion recognition. The above comparative analysis shows that the PSD-GAN data augmentation method proposed by us can significantly improve the EEG emotion recognition rate, and the frequency band correlation model is better than the frequency band separation model. This section discusses several noteworthy issues.

Firstly, we can see from the experiments of the DEAP dataset and MAHNOB-HCI dataset that the recognition accuracy has been significantly improved before and after data augmentation. We believe that there are two main reasons for the improvement of accuracy. On the one hand, the data augmentation increases the number of samples, and on the other hand, the data augmentation method we adopt increases the sample size of each category to the same, so the balance between categories is achieved. Therefore, the model can better learn the features between different categories, to reduce overfitting, improve generalization ability, and achieve a higher recognition rate.

Second, we can find that FBCCNN is always better than FBSCNN. In Figure 5, we can see the difference between the two network structures, which is mainly reflected in the different input methods. FBCCNN input is the overall input of four frequency bands to the convolution network. The FBSCNN input is that four frequency bands are input to the convolution network separately, and the features of the four frequency bands are integrated into the final full connection layer. Because of the characteristics of the convolutional neural network, we can know that FBSCNN can only extract the features of each frequency band, while FBCCNN can not only extract the features of individual frequency bands but also extract the features between frequency bands. Therefore, we can find that the correlation between frequency bands has an important impact on EEG emotion recognition. This correlation may be that the positive correlation of some features in band *θ* and band *α* is the expression of negative emotion, or the negative correlation of some characteristics in band *θ* and band *γ* is the expression of positive emotion.

Finally, the data augmentation method proposed by us can effectively improve the accuracy of the model. Through the comparative experiments of frequency band correlation and frequency band separation models, it is found that there are some correlation features between frequency bands, which can improve the model recognition rate, but there are still some problems that need to be further considered. For example, PSD-GAN network training is difficult and the quality of generated samples is unstable. In addition, what frequency band correlation features can effectively improve the recognition rate has not been revealed. Therefore, in the future, we will try to establish more stable and high-quality generation adversarial networks and strive to reveal the correlation features of key frequency bands to improve the recognition rate.

## 6. Conclusions

The work of this paper mainly includes two aspects. First of all, we propose the generative adversarial network PSD-GAN based on GAN to generate samples with PSD features. The proposed method of generating samples is of great significance to solve the problem of insufficient samples and imbalance of samples in the field of EEG recognition, and the samples generated by PSD-GAN greatly improve the accuracy of EEG emotion recognition. In the future, we will also consider other data expansion methods, such as transfer learning, migrating samples of other datasets, or network model parameters to achieve a high recognition rate. Secondly, we designed two different models, FBCCNN and FBSCNN, to explore the influence of frequency band correlation features on EEG emotion recognition. The final experimental results show that the FBCCNN that can extract the frequency band correlation feature is better than the FBSCNN that cannot extract the frequency band correlation feature in the EEG emotion recognition task. From this, we can conclude that the frequency band correlation feature has an important influence on the EEG emotion recognition task. This will provide a reference for future researchers in the design of neural networks.

## Figures and Tables

**Figure 1:** Constructing the 2D plane.

**Figure 2:** Flowchart of data processing. Due to space constraints, only 5 dimensions were drawn in the PSD column vector diagram, but actually it was 32 dimensions.

**Figure 3:** PSD-GAN structure.

**Figure 4:** Emotion classification model. In the above model, the value of *N* is 4, which represents the number of input bands (*θ*, *α*, *β*, and *γ*).

**Figure 5:** Performance comparison between relevant approaches.

**Table 1:** DEAP dataset general description.

Overall					
Subjects	Video	Channels	Sampling rate	Rating scale	Rating values
32	40	32	128 Hz	Arousal valence	Continuous scale of 1-9

**Table 2:** DEAP dataset subject description.

Subject		
Array	Array shape	Array content
Data	40 × 32 × 8064 (384 base + 7680 trial)	Video/trial × channels × data
Labels	40 × 32	Video/trial × label (valence, arousal)

**Table 3:** EEG patterns and corresponding characters.

Patterns	Frequency	Brain state	Awareness
Delta (*δ*)	1-3 Hz	Deep sleep pattern	Lower
Theta (*θ*)	4-7 Hz	Light sleep pattern	Low
Alpha (*α*)	8-13 Hz	Closing the eyes, relax state	Medium
Beta (*β*)	14-30 Hz	Active thinking, focus, high alert, anxious	High
Gamma (*γ*)	31-50 Hz	During cross-modal sensory processing	Higher

**Table 4:** Comparison of the number of two-category labels for arousal and valence before and after PSD-GAN data augmentation.

Subject	Data distribution before PSD-GAN				Data distribution after PSD-GAN			
	Arousal		Valence		Arousal		Valence	
	High	Low	High	Low	High	Low	High	Low
S01	1219	811	965	1065	1219	1219	1065	1065
S02	1218	812	1268	762	1218	1218	1268	1268
S04	1218	812	812	1218	1218	1218	1218	1218
S06	862	1168	1522	508	1168	1168	1522	1522
S07	1271	759	1421	609	1271	1271	1421	1421
S08	1218	812	1117	913	1218	1218	1117	1117
S09	1272	758	1066	964	1272	1272	1066	1066
S10	1116	914	1016	1014	1116	1116	1016	1016
S11	1269	761	1217	813	1269	1269	1217	1217
S17	1268	762	1118	912	1268	1268	1118	1118
S18	1269	761	1321	709	1269	1269	1321	1321
S22	1270	760	1015	1015	1270	1270	1015	1015

**Table 5:** Comparison of the number of labels in the four categories of valence and arousal before and after PSD-GAN data augmentation.

Subject	Data distribution before PSD-GAN				Data distribution after PSD-GAN			
	LVLA	HVLA	LVHA	HVHA	LVLA	HVLA	LVHA	HVHA
S01	506	305	559	660	660	660	660	660
S02	509	303	405	813	813	813	813	813
S04	557	1067	355	51	1067	1067	1067	1067
S06	306	862	202	660	862	862	862	862
S07	254	505	355	916	916	916	916	916
S08	457	406	456	711	711	711	711	711
S09	557	252	458	763	763	763	763	763
S10	456	458	558	558	558	558	558	558
S11	508	761	305	456	761	761	761	761
S17	355	457	557	661	661	661	661	661
S18	405	356	406	863	863	863	863	863
S22	508	303	609	610	610	610	610	610

**Table 6:** The recognition accuracy (%) of the two models in two classification tasks before and after data augmentation.

Subject	Case 1				Case 2			
	Valence		Arousal		Valence		Arousal	
	FBCCNN	FBSCNN	FBCCNN	FBSCNN	FBCCNN	FBSCNN	FBCCNN	FBSCNN
S01	86.04	82.67	86.43	83.16	90.83	89.25	92.25	89.09
S02	77.34	63.15	77.73	63.64	81.36	71.08	82.78	70.92
S04	80.44	62.44	80.83	62.94	85.13	72.39	86.55	72.24
S06	76.65	63.15	77.04	63.64	80.33	70.77	80.75	70.61
S07	90.10	70.05	88.49	70.54	95.10	80.19	95.52	80.03
S08	83.55	75.56	83.94	76.05	87.5	82.11	88.92	81.95
S09	84.58	73.84	84.97	74.33	89.86	79.94	90.28	79.78
S10	86.31	77.29	86.70	77.78	93.67	83.41	94.09	83.25
S11	80.10	66.60	80.49	67.09	86.16	75.89	87.58	75.74
S17	81.82	73.84	82.21	74.33	85.81	79.55	88.23	79.39
S18	79.41	66.94	79.80	67.43	86.05	73.86	87.47	73.70
S22	69.01	66.42	69.40	64.91	76.61	72.10	79.03	71.94
Average recognition accuracy results across subjects on “valence” and “arousal”								
Across subjects	82.40	78.65	83.55	77.15	88.90	83.64	90.26	80.55

**Table 7:** The recognition accuracy (%) of the two models in four classification tasks before and after data augmentation.

Subject	Case 1		Case 2	
	FBCCNN	FBSCNN	FBCCNN	FBSCNN
S01	65.08	59.23	76.00	68.87
S02	66.23	60.38	77.16	70.02
S04	59.64	53.79	70.57	63.43
S06	60.10	57.46	71.03	67.10
S07	60.86	55.01	71.78	64.65
S08	66.43	60.58	77.36	70.22
S09	64.90	59.05	75.83	68.69
S10	65.34	59.49	76.27	69.13
S11	66.22	60.37	77.15	70.00
S17	70.18	64.33	81.11	73.97
S18	58.06	52.21	68.99	61.85
S22	60.32	54.47	71.25	64.11
Average recognition accuracy results across subjects				
Across subjects	55.87	52.34	70.34	66.90

**Table 8:** Comparison results of the recognition rate before and after data augmentation.

	Data distribution before PSD-GAN			Data distribution after PSD-GAN		
	Negative	Neutral	Positive	Negative	Neutral	Positive
Number of samples	150	166	104	166	166	166
Average recognition accuracy (%)						
	Case 1			Case 2		
FBCCNN	62.06			70.34		
FBSCNN	56.78			66.50		

## Data Availability

The DEAP dataset data supporting this META-ANALYSIS are from previously reported studies and datasets, which have been cited. The processed data are available (https://github.com/panbo-bridge/eeg-emotion-recognition-base-gan-and-cnn/tree/master).
